The article "Investigation on Depression of College Students Majoring in Physical Education and Nonphysical Education: A StudyBased on the Age Region and Gender of 374 Students" was retracted in 2023. Reasons: signs of a paper mill; suspected computer-generated content; unreliable results or conclusions; lack of ethics approval or compliance.

# Investigation on Depression of College Students Majoring in Physical Education and Nonphysical Education: A StudyBased on the Age Region and Gender of 374 Students

**DOI:** 10.1155/2022/9106594

**Published:** 2022-09-02

**Authors:** Xiaofen Ding, Nian Tang

**Affiliations:** ^1^School of Physical Education, Hunan First Normal University, Changsha 410205, Hunan, China; ^2^College of Physical Education, Huzhou University, Huzhou 314000, Zhejiang, China

## Abstract

In the research on the relationship between depression and college students' major, there are some differences in the degree of depression between sports major and nonsports major students. Based on these results, we assume that there is the possibility of emotional differences between professional and nonprofessional sports. A total of 374 samples of students majoring in physical education and nonphysical education at the same university were analyzed by using the methods of literature review and data analysis. A total of 188 subjects, including 121 males and 253 females (186 majoring in sports and nonsports), were asked to fill in the SDS (Self-Rating Depression Scale). SDS is widely used in rough screening, emotional state evaluation, investigation, and scientific research of outpatients in clinical psychology departments. The research obtained the difference in depression degree in the whole sample and further compared the depression degree of students of different ages and native places. Statistical analysis was performed on all data using SPSS 23.0 software. Basic data description, paired chi-square analysis, and covariance analysis were used. The results show that in this sample, the maximum value (minimum/maximum value) of one item of the total depression score of nonphysical education students exceeds the average value by 3 standard deviations, and this shows that the general level of depression scores of non-PE majors is high; most non-PE majors are in mild depression, which is equal to the number of PE majors who are in a normal mood; and nonsports majors in cities are more likely to have mild depression.

## 1. Introduction

Depression has become a more prevalent mental illness than many people imagine [1], with core symptoms of marked and persistent sadness [2], loss of interest, and lack of energy [3]. Suicide is one of the most serious consequences for people with depression and has become the second leading cause of death among young people aged 15–29 years [4, 5]. The population at this age, most of which are in the student stage, especially college students, is the main component [6].

College students with depression usually felt hopeless and helpless [7], and adverse childhood experiences (ACEs) were recognized as long-distance risks of depression in adulthood [8, 9]; smartphone addiction [10, 11] and epidemic [12, 13]are also important causes of depression among college students, depression and race of college students [14], gender [15], and professional [16, 17].

The article "Investigation on Depression of College Students Majoring in Physical Education and Nonphysical Education: A StudyBased on the Age Region and Gender of 374 Students" was retracted in 2023. Reasons: signs of a paper mill; suspected computer-generated content; unreliable results or conclusions; lack of ethics approval or compliance.

A cross-sectional study has been widely used in studies related to depression and college students' majors [18–20]. There is a difference in the degree of depression between sports majors and nonsports majors. The incidence of depression among nonsports majors is significantly higher than that of sports majors [21]. Students who major in physical education are active, enthusiastic, and energetic. Regular physical exercise can effectively reduce the risk of depression [22]. Physical exercise and suicide behavior were negatively correlated, and the frequency of physical exercise had the greatest effect, followed by the duration and intensity of physical exercise [23].

Compared with college students who do not often engage in sports dancing, college students who often practice sports dancing are less prone to depression [24]. The combination of life and death education (LDE) and dance exercise therapy (DMT) can prevent and relieve depression in college students. We assume that there is the possibility of emotional differences between professional and nonprofessional sports. In the study of the relationship between depression and college students' major, there is a certain difference in the degree of depression between sports major and nonsports major students. On this basis, using the method of literature and data analysis, the paper analyzes the sample of 374 sports and nonsports major students at the same university. A total of 188 subjects, including 121 males and 253 females (186 sports and nonsports majors), were required to fill in the SDS. SDS is widely used in screening, emotional state evaluation, investigation, and scientific research of outpatients in clinical psychology departments. The study revealed differences in depression levels across the sample and further compared the levels of depression among students of different ages and origins.

## 2. Objective and Methods

### 2.1. General Description

A total of 374 college students (121 males and 253 females, including 186 PE majors and 188 non-PE majors) in Hunan First Normal University were investigated using the self-rating depression scale (SDS). We will publish the questionnaire online, please fill in the questionnaire at the link. A total of 488 copies were received. After screening, the anonymous questionnaire that was filled in less than one minute was deleted, and 374 people remained. SDS has been widely used in clinical psychology all over the world. After more than 20 years of localized revision in China, it has been applied to the rough screening of outpatients in clinical psychology departments, as well as the assessment and general investigation of adult emotional states, and has also been widely used in scientific research.

The article "Investigation on Depression of College Students Majoring in Physical Education and Nonphysical Education: A StudyBased on the Age Region and Gender of 374 Students" was retracted in 2023. Reasons: signs of a paper mill; suspected computer-generated content; unreliable results or conclusions; lack of ethics approval or compliance.

### 2.2. Statistical Analysis

Statistical analysis was performed on all data using SPSS 23.0 software. Basic data description, paired chi-square analysis, and covariance analysis were used.

## 3. Results and Discussion

Table 1 provides the analysis of the basic situation of PE major students and non-PE major students, including the students' native place and gender. Table 1 shows that more than 50% of the samples are “rural” in terms of the native regions of PE students. In addition, the proportion of urban samples is 41.40%. The proportion of “female” in the sample was 57.53%. The proportion of male samples was 42.47%. From the perspective of non-PE major students' native regions, more than 50% of the samples are “rural.” The proportion of urban samples is 44.15%. The proportion of “women” is 77.66%.

All the samples were investigated with Zun's depression questionnaire, and the scores were calculated. Describe the overall situation of the data according to the mean or median of two groups: PE students and non-PE students. It could be seen from Table 2 that the maximum value of the total depression score of non-PE majors in one item exceeded the average value by 3 standard deviations, indicating that the data fluctuated greatly. Compared with the average value, the median was more suitable for describing the overall level. The maximum (minimum/maximum) of the total depression scores of non-PE majors in one item of data exceeded the average by 3 standard deviations. This indicates that the overall level of the depression total score of non-PE major students is higher.

According to the results of the Chinese norm, the demarcation value of the SDS standard score was 53 points, of which 53–62 points were classified as mild depression, 63–72 points as moderate depression, and above 73 points as severe depression. The sample score is judged according to the standard.

Table 3 shows that the paired chi-square test is used to study the relationship between depression of PE major students and depression of non-PE major students. The number of categories compared in this pair was greater than 2 (i.e., paired multiclass), and therefore, the study was conducted using the Bowker test. Significant differences between paired data at the 0.05 level (chi = 178.103, *p* ≤ 0.001 < 0.05) were noted. The mild depression of non-PE majors was the same as the normal mood of PE majors, as shown in Table 4.

The article "Investigation on Depression of College Students Majoring in Physical Education and Nonphysical Education: A StudyBased on the Age Region and Gender of 374 Students" was retracted in 2023. Reasons: signs of a paper mill; suspected computer-generated content; unreliable results or conclusions; lack of ethics approval or compliance.

This study explored the correlation between milder depressive emotions presented by nonphysical education majors and “region of origin” and “gender.” Considering the potential interfering factors, the influence of “native place” on “depressed mood” and “age” and “gender” was likely to be the influencing factor, belonging to the interfering items. Therefore, it needs to be taken into account in the analysis. After analysis, the term of “gender” has no relationship with the term of “native place” for the term of “depressed mood,” so it was excluded. We used covariance analysis, and the interference term, also known as the “covariate,” is here the “age” term.

Table 5 shows the results of the parallelism test. In this case, only the significance of the interaction items should be concerned. The “Native area of non-PE major students ^*∗*^ age of non-PE major students” in the table was the interaction term of independent variable *x* and covariate. The data results showed that through the parallelism test (*F* = 0.041, *P*=0.072 > 0.05), the premise assumption of covariance analysis was met, and thus, it indicated that covariance analysis could be further conducted.

Table 6 shows the results of the covariance analysis. The square value of *R* in the above table is 0.005, which means that the native place and geographical source of non-PE students can explain 0.5% of the mild depression of non-PE students. Further expand the mean comparison of native regions to get Table 7.

Table 7 shows that the average depression score of the sample of non-PE major from rural areas is 48.21, which is less than 49.07 of the urban groups, indicating that in this sample, the urban non-PE major students are more prone to mild depression.

## 4. Conclusions

In this sample, the following conclusions are made:

1. The maximum (minimum/maximum) of the total depression score of non-PE students exceeds the average by 3 standard deviations. This indicates that the overall level of the depression total score of non-PE major students is higher.
2. Most of the nonphysical education students were in mild depression, and the number of these nonphysical education students was the same as that of the normal students.
3. Urban non-PE majors were more likely to have mild depression.

## 5. Discussion

We assume that there is the possibility of emotional differences between students majoring in physical education and nonphysical education majors. In the study of the relationship between depression and college students' majors, there are some differences in the degree of depression between physical education majors and nonphysical education majors.

The article "Investigation on Depression of College Students Majoring in Physical Education and Nonphysical Education: A StudyBased on the Age Region and Gender of 374 Students" was retracted in 2023. Reasons: signs of a paper mill; suspected computer-generated content; unreliable results or conclusions; lack of ethics approval or compliance.

Obviously, the innovation of the research still needs to be improved. As a cross-sectional study, we only discussed the situation of a sample in a university. In this sample, most of the nonphysical education majors were in mild depression, and the number of these nonphysical education majors was the same as those in normal mood. This may be due to significant data bias. Because there are twice as many women as men in this sample, and in a previous 17-year-old study of depression among Chinese college students, women were more likely to be depressed [25], so there is such a significant difference.

It should also be noted that urban non-PE majors were more likely to have mild depression. This is inconsistent with the existing research reports in academic circles in China and Western countries [26, 27]. Previous studies found that rural college students were more likely to commit suicide, and depression was the root cause of suicide. The reason for this is that we may use a cross-sectional design, and the sample size is too small for our student sample to represent the sample of college students from other universities in China. We cannot exclude unmeasured confounding factors at this time. The sample size can be further expanded in future studies to explore the reasons for this situation.

## Figures and Tables

**Table 1:** Basic information.

Name	Option	Frequency	Percentage (%)
Native place of sports major students (*n* = 186)	Rural area	109	58.60
	Urban area	77	41.40

Sports major student gender (*n* = 186)	Woman	107	57.53
	Man	79	42.47

Native place of non-PE major students (*n* = 188)	Rural area	105	55.85
	Urban area	83	44.15

Gender of non-PE major students (*n* = 188)	Woman	146	77.66
	Man	42	22.34

**Table 2:** Basic indicators.

Name	Sample size	Minimum value	Maximum	Average value	Standard deviation	Median
Total depression score of physical education major students	186	20.000	60.000	39.828	9.017	39.000
Total depression score of nonphysical education major students	188	27.000	79.000	48.590	6.417	48.000

**Table 3:** Paired chi-square analysis results.

match	Name	Depression among nonphysical education major students			Amount to	*χ* ^2^	*P*
		Moderate depression	Normal	Mild depression			
Depression of physical education major students	Normal	0	153	18	171	178.103	≤0.001^∗∗^
	Mild depression	2	0	13	15		
	Moderate depression	0	0	0	0		

Amount to	2	153	31	186	—	—	—

^*∗*^ *p* < 0.05. ^*∗∗*^*p* < 0.01.

**Table 4:** Comparison of depression among PE majors and non-PE majors.

	Depression of physical education major students		Depression among nonphysical education major students	
	*n*	Percentage	*n*	Percentage
Normal	171	91.94	2	1.08
Mild depression	15	8.06	153	82.26
Moderate depression	0	0.00	31	16.67
Summarize	186	100.00	186	100.00

The article "Investigation on Depression of College Students Majoring in Physical Education and Nonphysical Education: A StudyBased on the Age Region and Gender of 374 Students" was retracted in 2023. Reasons: signs of a paper mill; suspected computer-generated content; unreliable results or conclusions; lack of ethics approval or compliance.

**Table 5:** Parallelism test of covariance analysis.

Difference source	Sum of squares	*df*	Mean square	*F*	*P*
Intercept	3041.268	One	3041.268	74.385	≤0.001^∗∗^
Area of origin of non-PE major students	122.760	One	122.760	3.003	0.085
Age of non-PE major students	1.673	One	1.673	0.041	0.840
Area of origin of non-PE major students *∗* age of non-PE major students	134.245	One	134.245	3.283	0.072
Residual	7522.915	184	40.885		

*R* ^2^, 0.023. ^*∗*^*p* < 0.05.^*∗∗*^*p* < 0.01.

**Table 6:** Covariance analysis results.

Difference source	Sum of squares	*df*	Mean square	*F*	*P*
Intercept	3881.870	One	3881.870	93.788	≤0.001^∗∗^
Area of origin of non-PE major students	29.152	One	29.152	0.704	0.402
Age of non-PE major students	7.797	One	7.797	0.188	0.665
Residual	7657.160	185	41.390		

*R* ^2^, 0.005. ^*∗*^*p* < 0.05.^*∗∗*^*p* < 0.01.

**Table 7:** Native areas of non-PE major students.

Item	Average value	Standard deviation	*n*
Rural area	48.21	7.08	105
Urban area	49.07	5.47	83

## Data Availability

The data used to support the findings of this study are included within the supplementary file.

## Supplementary Materials

Supplementary Materials Raw data for the analysis.
